The article "Rural Planning Evaluation Based on Artificial Neural Network" was retracted in 2023. Reasons: unreliable results or conclusions; concerns about the data; concerns about the peer review; concerns about the citations.

# Rural Planning Evaluation Based on Artificial Neural Network

**DOI:** 10.1155/2022/9746362

**Published:** 2022-06-11

**Authors:** Yumei Liu, Xuezhou Huang

**Affiliations:** ^1^School of Geography Science and Geomatics Engineering, Suzhou University of Science and Technology, Suzhou 215009, China; ^2^Institute of Suzhou's Rural Revitalization Research, Suzhou 215009, China

## Abstract

The continuation of human civilization is inseparable from the development and construction of rural areas, and infrastructure is the core of rural development. China has been building large-scale rural infrastructure in recent years. Rural infrastructure building, for example, is huge in both quantity and scope, but it is beset by challenges in its current construction and development, and it urgently requires suitable leadership. Planning assessment, as a technical method, can identify problems in regional development and is a powerful tool for evaluating the impact of planning and construction and promoting the development of complete new areas. This paper is aimed at the planning evaluation of rural construction and the evaluation of rural construction and guides the planning and implementation of the next step of rural construction, to assist China's supervision and inspection of rural construction effect and promote rural construction and development into a good track. In view of the low accuracy and efficiency of the current evaluation model of rural planning and the problem that a single neural network easily produces local extreme value, the neural network method is improved, and the application of LM-BP neural network in the evaluation model of rural planning is proposed. Input sample elements are five factors affecting rural construction, including industrial construction, population distribution, and utilization rate of large-scale facilities, construction of public facilities, and promotion effect of supporting policies. Output sample is the evaluation result. On this foundation, the LM-BP neural network was used to convert the training into a least square problem, and the LM method was used to redefine the number of hidden layer nodes, resulting in the construction of a rural planning evaluation model based on the LM-BP neural network. This approach is used to determine the outcomes of rural planning evaluations. The experimental results show that the designed evaluation model has a small evaluation error, has the advantage of high accuracy compared with similar models, and is a reliable evaluation model for rural planning.

## 1. Introduction

In the process of realization after reform and opening up, the Central Work Conference discussed the “new normal” at the end of 2014, pointing out the direction of China's future progress. The new normal emphasizes the innovation of GDP growth mode, believing that the fundamental significance lies in meeting the actual needs of human material and cultural life, rather than merely pursuing quantitative growth. Reflected in urban and rural planning, the new normal emphasizes the characteristics of conforming to social development and focusing on quality rather than quantity [1]. In the past ten years, for the development and the rural demand level, urban and rural planning and construction of our country will focus on material space level; a large number of new area development, park construction, and large-scale and high strength facilities, beyond the living demand of residential development, emerge in endlessly; the focus of the urban and rural planning and construction shall be transferred accordingly; no need to pay attention to the growth of construction quantity. It requires control over the effectiveness and quality of construction. Instead of paying attention to the actual effect and profit of development and construction in the past, we should think about the rationality of planning and supervise and consider the implementation of planning.

Urban and rural planning evaluation started late in China, the theoretical basis is relatively weak, technology and methods are not yet mature, and the research has focused on the overall plan level, with single evaluation type; the characteristic of the large arbitrariness, its theoretical research, and practice to a certain extent is disjointed, before the urban and rural planning act was issued, and there are no supervision and related legal requirements [2]. Under the new situation, China's planning evaluation needs to be developed urgently, and relevant theories and mechanism construction need to be improved to ensure that the effectiveness and quality of construction are controlled in the whole process of planning and implementation and play a good driving role in rural development.

As a new rural space, the development of rural new areas will inevitably encounter various problems and obstacles, especially the comprehensive new areas with complicated functions. Harbin New Area was planned in 1990 and started construction in 2000, but the development level is still not high due to the high threshold of crossing the river. New Area was founded in 2001, and the permanent population of New Area was only 300,000 in 2011, which was quite short of the planned target of 1.5 million. With the continuous increase of rural new areas, the problem of building without city and city without employment in rural new areas is becoming more and more serious, and the phenomenon of “ghost city” emerges in endlessly [3]. The reasons are worth pondering. Is it the original site selection, positioning, land use planning, and other planning problems, or is there insufficiency in the implementation process? Faced with several issues in the development bottleneck, China's comprehensive rural new areas must find appropriate countermeasures, supervise the compilation and execution of appropriate planning, revise and adapt the development direction and mode, and get through the current bottleneck phase.

“To evaluate” means to appraise and measure. Referring to the explanation in Ci Hai, “evaluation” includes two basic processes: “measuring and evaluating the value of things” and “making general inferences about the nature, quantity, and change of things based on the current situation.” The Chinese “Evaluation” directly corresponds to English words such as Evaluation, Assessment, and Appraisal, which have different applications according to different contexts [4]. Among them, Evaluation is the most commonly used word to express the concept of Evaluation in western countries. Its etymology comes from “Value,” which is an activity to judge the Value of people or things. The U.S. Department of State defines it as “a systematic information collection and analysis tool” that improves efficiency and provides decision makers with current and possible future information based on the characteristics and outcomes of programs, projects, and processes. Evaluation is often used as an English explanation in the studies of planning Evaluation by domestic scholars [5]. Reasonable evaluation of rural construction can provide powerful data support for rural construction. As shown in Figure 1, the evaluation model can play a role in all aspects of rural planning. Therefore, it is crucial to find high-quality evaluation methods for rural planning.

There are many existing evaluation methods in China. Wei et al. [6] adopts the evaluation model of rural planning based on input-output analysis. From the input and output of buildings, the statistical data obtained from planning are relatively one-sided, leading to large errors in evaluation results. Liu et al. [7] proposed the loss assessment model based on maximum likelihood method, which easily falls into the state of local optimal solution, and the obtained assessment results have low credibility. Zhang et al. [8] uses the zoning classification method to evaluate the engineering planning and construction, starting from the factors that affect rural planning, in an attempt to fully grasp the situation of rural planning and accurately predict the evaluation results. However, because of overfitting in the training phase, this approach is prone to substantial errors in the evaluation outcomes. Hong-Juan conducted a preliminary study of the implementation evaluation of rural design [9] on the basis of emphasizing the importance of this evaluation. He drew important conclusions on the implementation level of rural design through an overall evaluation of the scope involved and an investigation of a typical case of a developed neighborhood. Planners can identify difficulties in the implementation process by conducting a rational review of rural design implementation. Taking the water supply special evaluation of new county as an example, Cheng et al. [10] evaluated the implementation results of the planning from three aspects of water source, water plant, and water distribution network and evaluated the main contents of the water supply special planning from the selection of water source, water consumption index, and daily variation coefficient. In the research method combining quantitative and qualitative methods, the evaluation results of each evaluation object are usually dimensionless in existing planning evaluation, and a group of results can be discussed under the same standard. Generally, three kinds of methods are used: grading evaluation, completion percentage calculation, and index deviation calculation. For example, in the comparative study method, the consistency between planning and construction implementation is usually compared, and the percentage of completion of each item is obtained according to land use classification, or the percentage of completion of major facility projects and the percentage of coverage of control regulations are obtained. For example, in the index system method, the effective degree of planning implementation is evaluated according to the grading evaluation method of “effective, general, and ineffective,” and then, the comprehensive score is weighted by combining the evaluation of the percentage of completion. The questionnaire survey principle uses the survey statistical results to make equal-weight statistics of “excellent, general, and poor” and uses the method of graded evaluation to get the final results [11]. Other studies compare the deviation between the current rural construction, social development, and other indicators and the planning and score according to the percentage of deviation between the current value and the target value.

Aimed at the problems of rural planning evaluation model and method, in this paper, the neural network was improved, because the state of a single neural network easily trapped in local minima and convergence for a long time; to obtain the optimal evaluation results, the design is based on LM-BP neural network assessment model; this model has two characteristics, one of which is on the basis of neural network. Converting network training into least square problem can solve the protracted problem of rural planning evaluation. Second, the number of iterations of LM-BP neural network training is limited to avoid training falling into local extremum state. Therefore, the model in this paper can ensure the accuracy of evaluation and improve the efficiency of evaluation. Simulation experiments are carried out to verify the efficiency evaluation effect, providing a reliable analysis basis for rural planning and construction.

The arrangements of the paper are as follows: Section 2 discusses the related work.  Section 3 discusses the algorithm design of the proposed work.  Section 4 examines the experiments and results.  Section 5 concludes the article.

## 2. Related Works

### 2.1. Current Situation of Rural Planning Evaluation

Western planning evaluation started in the 1950s, originated from the public policy evaluation of British and American countries, and experienced a process of transformation from rational planning to communicative planning in planning paradigm, from instrumental rationality to substantive rationality, and finally to communicative rationality. Based on these changes in the way of thinking, Guba and Lincoln [12] divides the evaluation into four stages from the value orientation in the fourth-generation evaluation: measurement, description, and judgment and value diversification [13]. In different stages, different viewpoints have emerged on the subject, object, and method of planning evaluation.

As for the subject of planning evaluation, Williams [14] distinguished each stage in the process of planning preparation and the relationship between evaluation executor and planner, as well as the time point of implementing evaluation and the specific content of evaluation. It is suggested that the evaluation criteria should be formulated by planners in the process of planning. As for the objects of planning evaluation, Kok et al. compared the development of planning evaluation and project evaluation at that time and believed that the evaluation before and during the implementation of planning evaluation had been marginalized [15]. De Oliveira et al. [16] takes a similar view, noting that there has been more research on preimplementation evaluations than on the implementation and postimplementation phases. In terms of planning evaluation methods, according to Guba's [12] four-generation classification method, western planning evaluation ideas and methods can be divided into four categories of “measurement-description-judgment-value diversification” in chronological order. According to their own characteristics, these methods can be used in different stages of planning and implementation. The first generation of evaluation, represented by the cost-benefit method proposed by Hill and Wehman [17], was first applied to public policy evaluation, which was “measurement” oriented evaluation. Based on the thinking mode of instrumental rationality, the currency is taken as the unit of measurement to determine the most stable operation mode, which is generally applied to the development activities of public undertakings and infrastructure construction. A similar method is cost-effectiveness analysis. The second generation of assessments introduces “descriptions” of things that cannot be directly quantified, in order to judge the consistency between the current situation and the described goals [18]. It tries to go beyond simple positivism and combine rational measurement with evaluation of target effectiveness. The representative methods are target realization matrix method and multiple index evaluation method, which decompose the total goal into multiple indexes, measure the target realization degree of each index through cost and income and then determine the overall goal realization situation through the weight of each index. The third generation of evaluation goes beyond pure rational planning and begins to consider the “judgment” of object value. It believes that the value orientation of evaluation is different, and the value judgment results of planning results are also diverse. Planning balance sheet and environmental impact assessment are both third-generation methods [19]. PBS method is a CBA method incorporating social analysis, considering the externality of the project. The fourth-generation assessment is based on the concept of communicative planning and is characterized by “value diversification,” emphasizing diverse participation, feasibility, and incremental development. Represented by the community impact analysis method proposed by Lichfield, it pursues a comprehensive, systematic, and composite analysis method.

The domestic research on planning evaluation started from the 1990s, and a series of related theoretical studies were carried out based on the western planning evaluation theory review. The focus is on the sorting and reference of relevant western theories and methods, the division of planning and evaluation stages, and the summary of research contents in each stage. Some scholars summarized relevant western theories in detail [20]. For example, Jenkins et al. [21] discussed the origin, theory, and content of modern planning evaluation in detail against the background of the mature planning evaluation system in the West. Song and Li [22] drew lessons from North American rural planning and evaluation experience and explored the development direction of planning and evaluation in China from the aspects of planning implementation subject, content of planning and evaluation, result expression, and public participation. Graymore et al. explored the planning evaluation methods in line with the development situation in China by sorting out the theoretical paradigms related to planning evaluation and the changing process of evaluation methods in western countries [23]. Represented by sun, domestic scholar's research content is more comprehensive; on the basis of summarizing the theories and methods of the western division of the type of planning evaluation, combined with its values and the paradigm shift, planning assessment and implementation effect evaluation put forward the corresponding ideas and methods and also stress the necessity and difficulty of planning evaluation research in China. Lu planning implementation evaluation can be divided into planning, planning, evaluation, planning, implementation, planning revision, and planning implementation after the completion of the five stages and put forward the measures for the rural planning and assessment of target oriented to promote rural planning form “compile-adjustment-evaluation” the virtuous circle, to cope with the problems in the planning and implementation stages. Through sorting out the planning time axis, McDonald et al. constructed a multiangle planning assessment model based on four factors, including technical means, planning objects, efficacy of the planning implementation stage, and postimplementation effect [24]. The special research of planning evaluation in “Overall Implementation and Technical Evaluation of Qingdao International Horticultural Expo Planning” suggests that the evaluation activities of rural planning should be discussed from three aspects: technical rationality, planning timeliness, and system coordination. In terms of technical rationality, it evaluates the scientific, feasibility, and rationality of the planning scheme from the aspects of environment, technology, and policy. In terms of planning effectiveness, the author examines the status quo of rural spatial development and the realization of rural spatial functions to judge whether planning can guide rural development. In terms of system coordination, short-term and long-term benefits, local and global benefits, and overall and group benefits of relevant planning should be considered to reflect their public policy attributes.

The western practice of planning evaluation is usually divided into three categories: planning preparation evaluation, planning implementation evaluation, and planning effect evaluation. As its name implies, it is divided according to the different evaluation objects of different stages of planning. Planning preparation evaluation is generally used to express whether the planning scheme or text is reasonable, and its practice is mostly targeted at specific special planning schemes, such as the quality evaluation of planning text of disaster prevention planning in the United States, the planning preparation action plan evaluation of New York low-carbon planning, and the planning preparation action plan evaluation of Auburn city. The primary purpose of the plan implementation evaluation is to track and monitor whether the plan is being implemented as planned and, in practice, to evaluate the regulations governing rural growth in the United States [25]. In general, systematic index evaluation or quantitative method is used to evaluate the planning effect within a certain range, such as Talen's [26] evaluation of the implementation of public facilities layout in Pueblo, Colorado, USA. In terms of the domestic situation, the classification of planning evaluation practice is usually based on the planning level, which mainly involves four levels: macro regional planning level, overall planning level, detailed planning level, special planning level, and other levels. After the promulgation of the Urban and Rural Planning Law and the measures, the number of relevant practical studies in China has increased significantly. Scholars have paid more attention to the level of rural master planning, while the number of evaluation studies on the level of detailed planning is relatively small. The Review and Countermeasures of Shenzhen Rural Master Planning in 2002 is an earlier research document with the meaning of planning evaluation in China, appearing in the form of “planning review.” At present, most of the research objects of planning evaluation practice in China are the villages at prefecture-level and above, and the evaluation methods are not systematic. Most of them are the evaluation after the implementation of planning, that is, the evaluation of planning implementation and the evaluation of planning effect.

### 2.2. Current Situation of Neural Network Evaluation Model

It was Banerji and Fisher [27], a statistician, who first put forward the classification problem of assessment in 1936. At that time, the assessment business in the United States began to develop and the business of many financial structures also developed rapidly. Financial institutions began to assess users' information in the process of processing application information, and expert system was the earliest system used for assessment. The system is used to evaluate applicants. In 1941, statistician Durand [28] used the characteristic dimension to assess the default risk of applicants, which was then used by financial institutions to distinguish between good and bad applicants. In 1996, Henley and Hand [29] applied the improved *K*-nearest neighbor method to financial risk assessment, which improved the prediction accuracy of data compared with the previous method. In 2003, Li et al. [30] used the linear discriminant method to predict the data, and the experiment proved that the classification tree has better results than other traditional methods. In 2005, Shi et al. [31] first used logistic regression to remove the features with high correlation and applied the results to artificial neural network to have better effect, so as to achieve the purpose of improving the effect of the model. In 2011, Buzius et al. [32] compared multiple classifiers through experimental research and carried out experiments on several commonly used classifiers. The results show that data modeling by machine learning has certain advantages, but it is still a complicated problem for classifier selection and model parameter tuning [33]. With the advent of the era of artificial intelligence, many scholars apply neural networks to evaluation models. In 2014, Oreski and Oreski [34] found that the data currently studied on financial institutions were all high-dimensional data, and too many irrelevant features might reduce the prediction accuracy of neural network. Oreski and Oreski [34] selects important features in data preprocessing through genetic algorithm and uses neural network modeling. In 2014, Fan et al. [35] used random forest as an evaluation model. Through experimental comparison, the model based on random forest has better generalization and prediction accuracy than the traditional single classifier model. Through the study of the literature, it was found that logistic regression and linear statistical method based on the current complex multidimensional nonlinear financial data have no good fitting effect; the traditional neural network to the dimensions of the data and data volumes have high requirements, such as random forests which also require a certain amount of data to get the ideal effect.

The standard particle swarm optimization algorithm is likely to have the same problem as gradient descent when solving space optimization; that is, particles trapped in local extremum cannot escape. Because each particle reduces the search space when exchanging information, it is possible that the particles still have a large space after convergent search. Many scholars' efforts in this area, such as adding iterative position changes in the late stage of the standard PSO algorithm, can enable particles with local convergence to jump out of the local optimal solution for global optimization. However, the effect of adding disturbed particles in the later stage is limited, because the earlier particles will quickly reduce the search range in the process of optimization. Some researchers increase the number of particles to cover a larger solution space and improve optimization outcomes. PSO, on the other hand, is still simple to fall into the local optimal solution as iteration times increase. The addition of genetic algorithm improves the possibility of searching global potential solutions, but its disadvantages are slow convergence rate and poor ability of searching local solutions.

Data is the basis of models. In planning evaluation, the security and privacy of data make it impossible to share data modeling, which is a limitation for the research in the field of evaluation models. In 2016, Google put forward the concept of federated learning, using the method of federated learning. In this application, the mobile phone, as the client participating in the modeling, trains the same model together under the coordination of the central server [36]. The author constructs a client-to-server architecture to protect data security, so that multiple clients can cooperate to train the model under the premise of ensuring data security. In addition, in recent years, there are many studies that combine federated learning with specific systems and combine federated learning with system functions to ensure the security of data involved in training. Therefore, for the evaluation problem, it is necessary to start from the algorithm model and data at the present stage. The algorithm model requires to ensure the ability of fitting complex data and find potential laws from high-dimensional nonlinear data, so as to achieve accurate prediction [37]. On the other hand, in view of the security and privacy of the data of financial institutions, the data quantity of the training model is increased through federated learning, and the data quality is indirectly improved, so as to improve the effect of the model.

## 3. Algorithm Design

In this section, we define the traditional assessment model and LM-BP neural network evaluation model in detail.

### 3.1. Traditional Assessment Model

Design evaluation model using the error backpropagation algorithm with more multilayer forward neural network (BP neural network), learning samples as input, and the corresponding expectations as output; the neural network weights and threshold depend on the realization and are expected to adjust the differential, the output value in line with expectations, and maximum output error sum of squares of the minimum [38]. Accordingly, the rural planning evaluation model based on neural network is constructed, as shown in Figure 2. In Figure 2, industrial construction, population distribution, utilization rate of large-scale facilities, construction of public facilities, and promotion effect of supporting policies are taken as input samples of the evaluation model.

Neural networks have strong adaptive capacity and higher level of generalization. Neural network was used to construct an evaluation model which can obtain more reliable evaluation result, but the state of single neural network is easily trapped in local minima and convergence when using long defects; to obtain the optimal evaluation results, the neural network is improved, and the evaluation model based on LM-BP neural network is obtained.

### 3.2. LM-BP Neural Network Evaluation Model

The LM algorithm is a nonlinear least squares method that uses a model function to evaluate parameter vectors using linear approximation. This step is finished in its field, and it changes network training into a least squares issue by ignoring derivative terms higher than bivalent. As a result, the LM-BP neural network can overcome the problem of classic neural networks' long convergence times. Based on the same sample capacity as a neural network, the LM-BP neural network is prone to falling into a local extremum state. This defect of LM-BP neural network can be avoided by setting the number of iterations. When the number of iterations of the LM-BP neural network reaches a certain limit, it is temporarily stopped. New weights and thresholds were assigned to the LM-BP neural network, and new iterative training was started until the desired results were obtained.

The contradiction between high training accuracy and a large number of training samples results in overfitting of the network and the reduction of network generalization ability [39]. The problem of decreased generalization ability can be solved by setting verification samples. In the process of verification sample training, if the sample accuracy decreases with the improvement of network accuracy, the network training should be terminated immediately. The training steps of the LM-BP neural network are described in Figure 3. When the training error does not meet the expected standard, the network training is reconducted until the sample training error meets the expected value, and the output model training results are obtained.

The LM-BP neural network evaluation model is designed. The number of input layer, hidden layer, and output layer is 1. The LM-BP evaluation model was trained using imitation software, and the number of hidden layer nodes was chosen to be 5 based on the findings of the optimal network training fitting [40]. The improved neural network evaluation model based on LM-BP is described in Figure 4.

In Figure 4, the five input nodes in the LM-BP neural network are industrial construction, population distribution, utilization rate of large-scale facilities, construction of public facilities, and promotion effect of supporting policies, and the last output node is the evaluation result. The weight matrix of LM-BP neural network from the input layer to hidden layer is described by *IW* {1, 1}, the threshold matrix is described by *B* {1}, the weight matrix from the hidden layer to output layer is described by *LW* {2, 1}, and the threshold matrix is described by *B* {2}.

Firstly, the correlation significance coefficient is obtained by using the following equation:

(1) $$\begin{array}{c} t_{nm}=\overset{p}{\underset{h=1}{\sum }}W_{nh}\frac{1-e^{-Wmh}}{1+e^{-Wmh}}. \end{array}$$

Secondly, equation (2) is used to obtain the correlation index:

(2) $$\begin{array}{c} T_{nm}=\left|\frac{1-e^{-tmh}}{1+e^{-tmh}}\right|. \end{array}$$

Finally, equation (3) is adopted to obtain the weight index of the evaluation index:

(3) $$\begin{array}{c} G_{nm}=\frac{T_{nm}}{\sum_{n=1}^{j}T_{nm}}. \end{array}$$

In the above formula, the input layer unit of LM-BP neural network is described by *i* and meets the conditions *n* = 1, 2, 3 ⋯ , *i*. The output layer unit of the LM-BP neural network is described by *m*, and *m* = 1. The weight value of the *h*th node of the hidden layer and the output layer of the improved LM-BP neural network is described by *m*_*h*_; the correlation significance coefficient and correlation index between the *n*_th_ input variable and the hidden layer are described by *t*_*nm*_ and *T*_*nm*_, respectively; and the influence of the *n*_th_ input variable on the evaluation result of the output is described by *g*_*nm*_. The neural network evaluation model based on LM-BP outputs the evaluation results. The LM-BP neural network rural planning evaluation model output evaluation results.

## 4. Experiments

In this chapter, we discuss the model prediction performance analysis and evaluating performance comparisons.

### 4.1. Model Prediction Performance Analysis

In order to verify the effectiveness of the proposed model in rural planning evaluation, a simulation experiment was carried out. The experimental sample is from the public data of rural planning evaluation in a certain region, and the sample records the data related to the construction and evaluation of the village from 2007 to 2016, with a total of 18 evaluations. 66% of the samples were used as training samples, 17% as testing samples, and the remaining 17% as verification samples. The scientific nature and reliability of the experiment can be assured after dimensionless processing of the experimental samples. If the sample error is set to increase for three consecutive times, the training will be stopped to prevent the faults produced by overfitting of the model in this paper. The model in this paper is used for sample training, and the weights of input variables on output variables are listed in Table 1.

The results are described in Figures 5 and 6, respectively.  Figure 5 describes the training errors of the model in the training samples, test samples, and verification samples. It can be seen from Figure 5 that before the experimental step number is 6, with the increase of the experimental step number, the error of the three samples of the model training in this paper gradually decreases and reaches the optimal state of the current training error when the step number is 6, which verifies the optimal point of the strong generalizing energy of the model in this paper. Between steps 6 and 9, the error of the validation sample increases continuously, which is consistent with the phenomenon that the model in this paper is prone to overfitting in the sample training process. During this process, the error of the training sample decreases gradually, while the error of the test sample increases gradually, which indicates that the model in this paper begins to overfit. Due to the relevant settings of the experiment to prevent overfitting, the experiment was stopped in time when the number of steps was 9, so as to avoid excessive error in sample training of the model in this paper, and the error of the training sample reached the target error value at this time.

Figure 6 shows the comparison between the predicted value and the actual value of the model in this paper. Figure 6 shows that the model prediction and the actual value are highly consistent; the abscissa describes the evaluation number of sample data and each assessment as a sample data, so the training samples for experiment 1~12 sample data confirm sample for 13~15 sample data, and prediction sample is 16~18 sample data. Figure 6 shows that the fitting degree of training and confirmation samples is good, and the actual value of data acquired from prediction samples is very consistent, based on this, which verifies the effectiveness and reliability of the model in this paper in rural planning evaluation.

In addition, the relative error of the evaluation results predicted by the model in this paper is described in Table 2. According to the data described in Table 2, with the progress of the test, the loss error of the model in this paper gradually decreases, and the error at the end of the experiment is only 0.85%, which can accurately achieve effective evaluation of rural planning.

### 4.2. Evaluating Performance Comparisons

To emphasize the model's benefits in this paper, a comparison experiment based on the input-output analysis and evaluation model was conducted, with data from a rural planning evaluation for 5 times or more from 2000 to 2018 chosen as the simulation experiment to increase the difficulty of sample training and planning evaluation and prediction. Industrial construction, population distribution, utilization rate of large-scale facilities, construction of public facilities, and promotion effect of supporting policies were taken as input variables of sample training, and planning evaluation was taken as output variables. Also, dimensionless operation was performed on experimental data to ensure the authenticity and reliability of experimental results.

The comparison between the evaluation results of the model in this paper and the evaluation model based on input-output analysis is listed in Table 3. As can be seen from Table 3, only in the third and seventh test, the evaluation error of the model in this paper is larger than 08%, which is 17.40% and 11.60%, respectively. The evaluation error of the model based on input-output analysis in these two tests is 13.40% and 18.70% higher than that of the model in this paper, respectively. In the other 5 tests, the evaluation error of the model in this paper is less than 06%, and in the sixth test, the error is the smallest, only 1.40%. At this time, the evaluation error of the model based on input-output analysis is 12.60%, much higher than that of the model in this paper. On the whole, the mean value of the evaluation error of the model in this paper is 5.60%, while that of the model based on input-output analysis is 8.90%, which is 6.70% higher than that of the model in this paper. Based on the above data, it can be seen that the model in this paper has high accuracy and small error in rural planning evaluation, so the evaluation performance of the model in this paper is better and has strong advantages compared with similar models.

The high evaluation accuracy of the model in this paper is because the model in this paper introduces LM algorithm on the basis of the single god meridian network and converts the network training into the least square problem. By setting the number of iterations, the LM-BP neural network is avoided to fall into the local extremum state, and the training accuracy of the model is improved.

## 5. Conclusions

This research presents an assessment model in light of the paucity of evaluation of rural planning in existing studies. A neural network evaluation model based on LM-BP is presented to increase the accuracy of rural planning evaluation. The model has three layers: input, hidden, and output. The five elements that influence rural planning are used as input samples, and estimation results are obtained via hidden layer learning. In this process, the model in this paper transforms the neural network training into the least square problem, which effectively shortens the network convergence time and improves the training efficiency, which is one of the characteristics of the model in this paper. At the same time, the model in this paper sets the iteration times of network training to avoid local extreme values of the LM-BP neural network. When the iteration times of LM-BP neural network training reach a fixed limit, the test is stopped, and new weights and thresholds are assigned to LM-BP neural network training to start new iterative training and stop when the desired results are obtained. This is another characteristic of the model in this paper. Through this step, the problem that the neural network easily falls into local extremum is solved. This methodology achieves efficient and accurate rural planning evaluation based on these two criteria. The findings demonstrate that this model's predicted value is nearly identical to the actual value, and it has a greater prediction accuracy than a similar model. This model meets the needs of planning evaluation in terms of evaluation accuracy and efficiency and provides scientific analysis basis for rural planning.

## Figures and Tables

**Figure 1:** Schematic diagram of the evaluation model applied to rural planning.

**Figure 2:** Neural network-based rural planning evaluation model.

**Figure 3:** Training steps of LM-BP neural network.

**Figure 4:** Improved neural network evaluation model based on LM-BP.

**Figure 5:** Comparison curves of training errors of three samples.

**Figure 6:** Comparison of predicted and actual values of the model in this paper.

**Table 1:** Influence weights of input variables on output variables.

Input variables	Weights
Industry construction	0.134
Population distribution	0.175
Utilization rate of large facilities	0.096
Public facility construction	0.186
Effect of supporting policies to promote	0.169

**Table 2:** Relative error of the prediction sample.

Relative error	Test sample output	Test sample target
10.26%	86.50	79.40
6.81%	83.60	75.10
2.57%	88.70	86.80
1.39%	90.40	89.40
0.85%	89.20	88.50

**Table 3:** Relative errors of the model in this paper compared with the traditional model.

True value	Our model results	Relative error	Input-output model results	Relative error
78.20	83.70	7.90%	62.50	14.20%
85.60	81.50	8.50%	59.70	16.10%
67.50	62.80	5.20%	84.90	12.50%
76.40	78.60	8.60%	91.40	13.30%
83.70	88.40	4.70%	95.3	10.70%
87.90	82.30	6.30%	71.20	9.50%
84.30	87.10	1.40%	73.50	12.70%
77.80	76.10	3.80%	87.20	8.70%

## Data Availability

The datasets used during the current study are available from the corresponding author on reasonable request.
